# Effect of coffee on color stability and surface roughness of newly introduced single shade resin composite materials

**DOI:** 10.1186/s12903-023-02942-y

**Published:** 2023-04-22

**Authors:** Shaimaa Rohym, Hossam El Mandouh Tawfeek, Raghda Kamh

**Affiliations:** 1 Conservative Dentistry, Al-Ahram Canadian University, Fourth Industrial Zones, Giza, Egypt; 2 Conservative Dentistry, Suez Canal University, Ismailia, Egypt; 3 Conservative Dentistry, Egyptian Russian University, Cairo, Egypt

**Keywords:** Single-shade composite resin, Color stability, Coffee, Surface roughness, Atomic Force Microscope, Profilometer

## Abstract

**Background:**

Dentists started to follow the era of using single-shade resin composite restorations to avoid color shade selection. Our study was done to evaluate and compare the color stability of two single-shade resin composite materials.

**Methods:**

Sixty samples were randomly allocated into two main groups (*n* = 30) according to the composite resin used: Group O: (Omnichroma) samples and Group V: (Venus Peral) samples. Each group was then divided into two subgroups (*n* = 15): group O1 and V1: samples immersed in coffee. Group O2 and V2: samples immersed in distilled water. Color changes (ΔE) and roughness values (Ra) were evaluated at baseline, first, and 14^th^ days of immersion. The color change was assessed using Vita Easyshade V, while surface roughness was assessed using a profilometer and Atomic Force Microscope (AFM). Data were collected and statistically analyzed using two-way variance analysis (ANOVA) and Tukey's post-hoc test (*p* < 0.05).

**Results:**

Group O1 and V1 recorded the highest ΔE_00_ (*P* = 0.002, 0.0001, respectively) and Ra values (*P* < 0.001) with no significant difference between both materials at 14 days.

**Conclusion:**

Single shade resin composite with innovative chromatic material technology has dramatic color change and surface roughness that sacrifice esthetic success.

## Background

Demand for ideal esthetic material in restoring teeth impacted both materials and techniques [1]. Dentists have recently preferred ceramic and resin-containing restorative materials [2] based on their esthetic and biological properties [3]. The Esthetic successes of dental resin composite restorations depend primarily on their surface properties and color stability.

Using nanotechnology in dentistry, manufacturers are now introducing resin composite materials with single-shade systems instead of more complex color systems. These materials have color harmony with tooth structure due to their nanofillers and nanocluster content. Recently, single-shade resin composite, which can be used for all tooth shades, has been introduced to the dentist's use. The advantage of its color-matching ability is that it eliminates the need for a shade-taking procedure. It reduces composite inventory, minimizing chair time for the patient and the wastage of unused composite shades [4].

Composite resins' color stability and surface roughness are essential for esthetic success [5]. Color changes have been associated with diet, chemical reactions, water absorption, and poor oral hygiene [5]. Consumption of certain beverages may affect the esthetic and physical properties of the resin composite, thereby destabilization the quality of restorations [6]. Beverages such as coffee, tea, cola, and wine cause different degrees of discoloration of resinous restorative materials [4]. It was reported that a surface roughness value below 0.15 μm. Decreases the adhesion of streptococcus mutans, while when this value is above 0.2 μm creates an accessible retention area for the attachment of the bacterial plaque [7].

In order to assess the color stability of restorative materials, many instrumental techniques could be used, such as; Digital cameras, Spectrophotometers, or colorimeters. Evaluating (ΔE) is referred to Commission International De L’éclairage (CIE) system [4].

Surface roughness is considered one of the reasons for exterior discoloration [8]. Wear of dental resin composites denoting debonding of inorganic fillers from the resin matrix, which leaves voids, increasing the surface roughness and forming a surface susceptible to exterior stain [8]. Mechanical and Optical profilometers, SEM (scanning electron microscope), and AFM (atomic force microscope) are widely used devices to measure and evaluate the surface roughness of restorative materials. Dental experts preferred profilometers as no preparation is required on samples to measure surface roughness, and repeated measurements are enabled [9]. Moreover, AFM obtains high-resolution 3D nanometric images for the material surface, offering complete surface quantification [10].

Our study examines the color stability and surface roughness of innovative chromatic resin composite after exposing them to commonly consumed beverages and coffee for 14 days using Vita Easyshade V, a contact stylus profilometer, and AFM. The null hypothesis was that there was no difference in the ΔE and Ra of both single-shade composite resins after immersing in coffee for 14 days.

## Materials and methods

### Materials

- Resin Composite Materials: (Omnichroma/Venus pearl) (Table 1)
- The beverages used were coffee (Nescafe classic, Nestle, Switzerland) and distilled water (Pharmapack, Egypt).

**Table 1:** Composition of the restorative materials used in this study

Product name	Type	Resin matrix	Filler average size	Filler volume	Filler weight	Product number	Manufacturer
Omnichroma	Supra-nano spherical	UDMA, TEGDMA	260 nm	68%	79%	1615	Tokuyama-Dental, Tokyo, Japan
Venus pearl	Nano-hybrid	TCD-DI-HEA UDMA, TEGDMA	5 nm – 5 μm	64%	76%	K010206	Kulzer GmbH, Germany

### Methods

#### Study design

Sixty samples were randomly allocated into two main groups (*n* = 30) according to the composite resin used. Group O: samples were obtained using single-shade composite resins (Omnichroma), and Group V: samples were obtained using single-shade composite resins (Venus Peral**)**. Each group was then divided into two subgroups (*n* = 15): group O1 and V1: samples immersed in coffee. Group O2 and V2: samples immersed in distilled water. The color change (ΔE) and roughness values (Ra) were evaluated for all samples at baseline (before immersion), and on the 1^st^, and 14^th^ days of immersion. Color assessments were measured using Vita Easyshade V, while surface roughness was measured using a contact stylus profilometer and AFM. The study proposal was reviewed and approved by the Research Ethics Committees (REC) of the Faculty of Dentistry, Cairo University, Egypt, on 29/3/2022. With approval number 30.3.22.

#### Sample size calculation

Sample size calculated depending on a previous study (Aydın et al.) [4] as reference. According to this study, the response within each subject group was normally distributed with a standard deviation of 1.4. If the actual difference in the experimental and control means is 1.8, the study minimally needed 11 subjects in each group to reject the null hypothesis that the population means of the experimental and control groups are equal with probability (power) 0.8. The type I error probability associated with this null hypothesis test is 0.05. The total sample size increased to 15 subjects per group to compensate 20% dropout.

#### Samples preparation

##### Resin composite specimens’ preparation

Thirty cylindrical disk-shaped specimens (6 mm diameter and 2 mm thickness) were prepared using a customized Teflon mold, rendering 60 specimens for the two resin composite materials. A Teflon mold and copper ring were fabricated with 2 mm thickness and 20 mm diameter with a centralized hole of (6 mm diameter and 2 mm thickness) in which the resin composite was bulk packed as one increment [4].

According to the manufacturer’s recommendations, the resin composite materials were dispensed, manipulated, and polymerized. A nylon thread was incorporated into the specimen before polymerization to allow their easy handling and their suspension in the immersion solutions during all aging periods. The resin composite was bulk packed inside the central hole of the split Teflon ring. To ensure that specimens would have flat polymerized surfaces free of bubble formation after curing, both top and bottom surfaces were covered with transparent polyester matrix strips (TOR VM, Moscow, Russia) and a microscopic glass slide (1 mm thickness) [4].

Specimens were polymerized for 20 s on both surfaces (top and bottom) using a light-emitting diode unit (LED COXO DB-686 MOCHA) through the glass slide and the polyester matrix strip. LED light curing unit was used in standardized mode, emitting 1200mW/cm2 irradiance as measured with a radiometer (Kerr manufacturing product). Then the two wings of the ring were opened to remove the specimens. The dimensions of the specimens were checked with a caliper (Pirmadent Germany SS). All samples were finished and polished using Sof-Lex disks (three-step system), starting with medium grit, then fine grit, and finally superfine grit, all in a dry media for 15 s. Then rinsing and drying with a water/air syringe for a total of 6 s [11]. Specimens were stored in distilled water in tight vials for 24 h at 37° C before the immersion procedures in the incubator [4].

##### Test solution preparation

With each type of resin composite, the 30 specimens were randomly allocated into two subgroups (*n*= 15 per subgroup), according to the immersion solution to be investigated. The two immersion solutions used were: distilled water (control solution) and coffee. The coffee solution was prepared by adding 3.6 g of coffee using a digital spoon scale to 300 ml distilled water, then boiling for 10 min to have a standardized concentration [12]. Filter paper was used to remove any impurities of the prepared coffee before being poured into vials and left to be cooled. Specimens were immersed through suspension with the nylon thread of 5 ml immersion solution. The immersion solutions were changed daily till the last assessment period. After placing specimens, the vial was sealed tightly with its cap to prevent any evaporation of the immersion solutions [4]. The containers were stored at 37 °C by placing them in a thermal control unit**.**After each storage period, the specimens were removed from immersion solutions and allowed to dry before color assessments. Then after assessments, the identical specimens were stored again in the vials containing daily fresh solutions for the following storage period [4].

##### Color measurements testing

Color shade assessment using Commission International de L’Eclainge (CIELab) color system (L*, a* and b* values) at baseline before immersion, after one day, and after 14 days by digital spectrometer device Vita Easyshade V (VITA Zahnfabrik, Bad Säckingen, Germany). It is a portable spectrophotometer and a new fifth generation of Easyshade with a handpiece of fiber optic probe assembly for illuminating and receiving the reflected light from the sample. Results appear through a LED screen. The base unit has the calibration block into which the handpiece is seated. The Easyshade handpiece has a 5 mm diameter stainless steel probe [13]. measurements by Vita Easyshade started with a calibration process that was performed per the manufacturer's instructions [13]. The probe was perpendicular to the recorded specimen before pressing the measurement on, and the results were displayed. According to the manufacturers’ instructions, two successive measurements were done and reported for each sample [13].

Color difference (ΔE^∗^_00_) values were calculated using the following formula CIEDE2000 for each specimen against white backgrounds [14]:

$${{\varvec{\Delta}}\mathbf{E}}_{00}\left({{\varvec{L}}}_{1}^{\boldsymbol{*}},\boldsymbol{ }\boldsymbol{ }{{\varvec{a}}}_{1}^{\boldsymbol{*}},\boldsymbol{ }\boldsymbol{ }{{\varvec{b}}}_{1}^{\boldsymbol{*}};\boldsymbol{ }{{\varvec{L}}}_{2}^{\boldsymbol{*}},\boldsymbol{ }{{\varvec{a}}}_{2}^{\boldsymbol{*}},\boldsymbol{ }{{\varvec{b}}}_{2}^{\boldsymbol{*}}\right)=\boldsymbol{ }{{\varvec{\Delta}}\mathbf{E}}_{00}^{12}={{\varvec{\Delta}}\mathbf{E}}_{00}$$

The L * value represents the lightness of an object where the value of zero equals a perfect black while the value of 100 represents a perfect reflecting diffuser. The a* value is a degree of redness of the color (positive a*; + 80) or its greenness (negative a*; − 80). Finally, the b* value counts for the degree of yellowness (positive b*; + 80) or its blueness (negative b*; − 80). The smaller the ΔE_00_, the lower the color change between the initial color measurement and the final color of the tooth. The perceptibility threshold (ΔE_00_) was 0.8 whereas the 50:50% acceptability threshold (ΔE_00_) was 1.8 [14].

##### Surface roughness testing

The surface roughness of the materials was tested using a contact stylus profilometer (SJ- 210 Surface roughness tester Mitutyoyo Japan). Each specimen was fitted to the specimen holder, where the surface was to be measured in the horizontal direction; then, the specimen holder moved in a vertical direction up to the specimen surface, touching the measuring tip. Device calibration is done according to the manufacturer's instructions before use https://www.mitutoyo.com/webfoo/wp-content/uploads/Surftest_SJ-210_310.pdf. Five readings were recorded for each specimen at a distance of 500 microns each.

Testing parameters:

1. Measuring distance 4 mm
2. Measuring Speed 0.5 mm/s. Returning 1 mm/s
3. Measuring force 0.75 mN
4. Stylus profile: tip radius 2-micron, tip angle 60 degree
5. Evaluation parameter Ra values expressed in microns

#### Surface morphology analysis using Atomic Force Microscope (AFM)

Surface morphology analysis was gained using the Atomic Force Microscope (Tosca 200 AFM—Anton Paar GmbH – Germany, tapping mode—500 um increment—rate 1 line/second) in 'contact' mode. Four regions were chosen to have different images which can be scanned by software (Mountains® 8.2 Software—Digital Surf, Besançon, France).

### Statistical analysis

All data were presented as mean &standard deviation. Data were presented in 1 table & 1 graph. Statistical analysis was performed with SPSS 16 ® (Statistical Package for Scientific Studies), Graph pad prism & windows excel.

The given data was extracted using the Shapiro–Wilk test and Kolmogorov–Smirnov test for normality, which revealed that the significant level (*P*-value) was insignificant as *P*-value > 0.05, which indicated that the alternative hypothesis was rejected. The concluded data originated from a normal distribution (parametric data) resembling a standard Bell curve.

## Results

### Color measurements results

#### Comparison between different materials

Comparison between different materials was performed by using the One Way ANOVA test, which revealed a significant difference between different groups after one day and after 14 days as *P* < 0.05, followed by Tukey’s Post Hoc test for multiple comparisons, which represented that after one day, V1 was significantly the highest color changes (17.09 ± 5.87), then O1 (12.46 ± 1.89), while there was insignificant difference between V2 (2.64 ± 0.86) and O2 (2.45 ± 1.40). After 14 days, V1 (26.94 ± 6.21) and then O1 (16.69 ± 3.52), while there was an insignificant difference between V2 (3.97 ± 0.67) and O2 (2.91 ± 1.30), as presented in Table 2 and Fig. 1.

**Table 2:** Mean & standard deviation of color changes (ΔE after one day and after 14)

Group	N	ΔE After 1 day		ΔE After 14 days		*P* value
		M	SD	M	SD	
**Omnichroma coffee O1**	15	12.46^a^	1.89	16.69^a^	3.52	0.002*
**Venus Peral Coffee V1**	15	17.09^b^	5.87	26.94^b^	6.21	0.0001*
**Omnichroma distilled water O2**	15	2.45^c^	1.40	2.91^c^	1.30	0.003*
**Venus Peral distilled water V2**	15	2.64^c^	0.86	3.97^c^	0.67	0.001*
***P*** ** value**		< 0.0001*		< 0.0001*		

*M* Mean, *SD* Standard deviation, *N* Count

^*^: Significant difference as *P* < 0.05

Means with the same superscript letters in the same column were insignificantly different as *P* > 0.05

Means with different superscript letters in the same column were significantly different as *P* < 0.05

^a^, ^b^ and ^c^ letters describes the significance determined by Turkey's post hoc test for multiple comparisons

**Fig. 1:** Bar chart representing color changes (ΔE after 1 day and after 14 days) in all groups

#### Comparison between color changes after one day and after 14 days

Comparison between ΔE after one day and after 14 days was performed using Paired t-test, which revealed a significant increase in color changes after 14 days in all groups, as presented in Table 2 and Fig. 1.

### Surface roughness results

#### Comparison between different intervals (effect of time) Table 3 and Fig. 2

**Table 3:** Descriptive statistics of all groups regarding surface roughness at baseline, after one day, and after 14 days and comparison between different intervals within each group

		**Min**	**Max**	**M**	**SD**	***P*** ** Value** **(One Way ANOVA test)**
**Omnichroma coffee** **O1**	**Baseline**	0.096	0.127	0.110^a^	0.010	< 0.0001*
	**After 1 day**	0.267	0.536	0.390^b^	0.090	
	**After 14 days**	0.238	0.760	0.530^c^	0.140	
**Venus Peral Coffee** **V1**	**Baseline**	0.011	0.429	0.260^a^	0.120	< 0.0001*
	**After 1 day**	0.333	0.646	0.491^b^	0.090	
	**After 14 days**	0.391	0.738	0.590^c^	0.090	
**Omnichroma distilled water** **O2**	**Baseline**	0.018	0.224	0.12^a^	0.060	< 0.0001*
	**After 1 day**	0.024	0.270	0.15^a^	0.080	
	**After 14 days**	0.148	0.503	0.303^b^	0.100	
**Venus Peral distilled water** **V2**	**Baseline**	0.009	0.390	0.231^a^	0.110	< 0.0001*
	**After 1 day**	0.034	0.483	0.240^a^	0.120	
	**After 14 days**	0.231	0.642	0.406^b^	0.120	

*Min* Minimum, *Max* Maximum, *M* Mean, *SD* Standard deviation

^*^Significant difference as *P* < 0.05

Means with different superscript letters were significantly different as *P* < 0.05

Means with the same superscript letters were insignificantly different as *P* > 0.05

^a^, ^b^ and ^c^ letters describes the significance determined by Turkey's post hoc test for multiple comparisons

**Fig. 2:** Line chart representing surface roughness changes in all groups

Comparison between different intervals was performed by using the One-Way ANOVA test, which revealed a significant difference in all groups as *P* < 0.05, followed by Tukey’s Post Hoc test for multiple comparisons, which revealed that:

- In Omnichroma coffee O1 and Venus Peral Coffee V1, there was a significant difference between all intervals (significant increase as all with different superscript letters)
- In Omnichroma distilled water O2 and Venus Peral distilled water V2 there was an insignificant difference between baseline and after one day, while after two weeks was significantly the highest.

## Comparisons between different groups Table 4 and Fig. 3

**Table 4:** Mean and standard deviation of roughness at baseline, after one day, and after 14 days and comparison between different groups

Group	N	Baseline		After 1 day		After 2 weeks	
		M	SD	M	SD	M	SD
**Omnichroma coffee** **O1**	15	0.11^a^	0.01	0.39^a^	0.09	0.53^a^	0.14
**Venus Peral Coffee** **V1**	15	0.26^b^	0.12	0.49^b^	0.09	0.59^a^	0.09
**Omnichroma distilled water** **O2**	15	0.12^a^	0.06	0.15^c^	0.08	0.303^b^	0.1
**Venus Peral distilled water V2**	15	0.23^b^	0.11	0.24^c^	0.12	0.406^b^	0.12
***P*** **value** **(One Way ANOVA)**		< 0.0001*		< 0.0001*		< 0.0001*	

*M* Mean, *SD* Standard deviation

^*^Significant difference as *P* < 0.05

Means with different superscript letters were significantly different as *P* < 0.05

Means with the same superscript letters were insignificantly different as *P* > 0.05

^a^, ^b^ and ^c^ letters describes the significance determined by Turkey's post hoc test for multiple comparisons

**Fig. 3:** Bar chart representing a comparison between all groups regarding surface roughness at all intervals

Comparison between different intervals was performed by using the One-Way ANOVA test, which revealed a significant difference in all groups as *P* < 0.05, followed by Tukey’s Post Hoc test for multiple comparisons, which revealed that:

- At baseline: Omnichroma coffee O1 and Omnichroma distilled water O2 were significantly the lowest with insignificant difference between them (same have letter a), while Venus Peral Coffee V1 and Venus Peral distilled water V2 was significantly the highest with insignificant difference between them (same have letter b).
- After one day: Omnichroma distilled water O2, Venus Peral distilled water V2 were significantly the lowest with insignificant difference between them (same have letter c), then Omnichroma coffee O1, while Venus Peral Coffee V2 was significantly the highest.
- After two weeks: Omnichroma coffee O1 and Venus Peral Coffee V1 were significantly the highest with insignificant difference between them (both have the letter a), while Omnichroma distilled water O2 and Venus Peral distilled water V2 were significantly the lowest with insignificant difference between them (same have letter b)

### Correlation between color changes and surface roughness

Correlation between surface roughness and color changes was calculated using Pearson`s Correlation Coefficient (r), which revealed a powerful (*r* > 0.8), positive ( +), significant (*P* < 0.05) correlation between them in both groups Table 5.

**Table 5:** Correlation between color changes (ΔE) and surface roughness after one day and after 14 days in both groups

Group	After 1 day		After 14 days	
	r	*P* value	r	*P* value
**Omnichroma coffee** **O1**	0.94	0.0001*	0.97	0.0001*
**Venus Peral Coffee** **V1**	0.95	0.0001*	0.96	0.0001*
**Omnichroma distilled water** **O2**	0.96	0.0001*	0.95	0.0001*
**Venus Peral distilled water V2**	0.95	0.0001*	0.97	0.0001*

### Atomic Force Microscope results

The surface roughness results measured by the contact stylus profilometer were explained and proved by the AFM analysis (Figs. 4, 5, 6 and 7).

**Fig. 4:** AFM photographs of the surface topography of Omnichroma resin composite group O1 (**a**) baseline (**b**) after 1-day immersion in coffee (**c**) after 14 days immersion in distilled water

**Fig. 5:** AFM photographs of the surface topography of Omnichroma resin composite group O2 (**a**) baseline (**b**) after 1-day immersion in distilled water (**c**) after 14 days immersion in coffee

**Fig. 6:** AFM photographs of the surface topography of Venus Pearl resin composite group V1 (**a**) baseline (**b**) after 1-day immersion in coffee (**c**) after 14 days immersion in coffee

**Fig. 7:** AFM photographs of the surface topography of Venus Pearl resin composite group V2 (**a**) baseline (**b**) after 1-day immersion in distilled water (**c**) after 14 days immersion in distilled water

## Discussion

The wide use of the shades of adhesive composite as esthetic restoration in anterior and posterior teeth paid attention to its multiple steps and the time consumption that posed challenges for dentists [15]. Recently, many manufacturers introduced a new single-shade resin composite as it has the advantage of reducing chair time and shade selection time [15]. Moreover, it was reported that any discoloration in the resin composite would affect the aesthetic [16, 17]. Hence, the current study presented the problems of color stability of resin composite after exposure to commonly consumed drinks of different storage periods. The null hypothesis in this study was rejected due to statistically significant differences in color and surface roughness values of both resin composite materials before and after immersion at evaluation with the Vita easy shade, profilometer, and AFM.

The color stability and surface characteristics of the two single-shade resin composites depend on the different compositions, fillers, particle size, and distributed resin matrix. A commercially available supra-nanofiller resin composite (omnichroma) was compared against a nanohybrid resin composite (Venus pearl). Nanotechnology applications introduced in the fillers size range within 0.1- 100 nm to improve properties [18]. Studies evaluating the stability of single structured resin composite severely need more to assert its chemical performance. It was stated that details of the fabrication conditions for the organic filler distributed inside the Omnichroma resin could be more precise [19].

The esthetic and mechanical properties of resin composite are influenced not only by their chemical composition but also by the environment to which they are exposed such as chemical agents found in saliva, foods, and beverages either intermittently or continuously. Coffee is an intense stain [4, 20], and a favorable drink used daily by most people. So, it was chosen as one of the experimental immersing solutions. While distilled water was used as a control to investigate the behavior of the resin composite itself [21]. It is worth mentioning that artificial saliva and distilled water have the same effect on resin composite [22].

In this study, each step was made to standardize the methodology; the specimens’ thickness of 2 mm for the light cure unit, and the curing time was adjusted to 40 s with 20 s exposure time for the top and 20 s for the bottom, respectively [23], miller strip and the standardized finishing and polishing procedures. Specimens were immersed in distilled water for 24 h before immersion in the tested solutions to complete polymerization [16].

In the current in-vitro study, a static immersion was done for all specimens for one day and 14 days, equivalent to one month and 14 months of consumption, respectively [16]. The increase in temperature will accelerate color change in the restoration [24]; specimens were incubated to adjust the temperature at 37°c all the storage time to simulate the oral environment. Coffee was replaced with a new proportion every 24 h to minimize bacterial growth. 

Visual perception of color is a psychological point-view and, unfortunately, depends on the observer's skill [21]. In order to overcome the problem of visual assessment of the color, many color-evaluating devices have been used as Colorimeters and Spectrophotometers that are more precise than the naked eye [21]. Color assessments in our study were done using a digital spectrometer device, Vita Easyshade V. This device is considered a reliable tool to measure the color change not only in clinical applications but also for research purposes in evaluating color interactions of human teeth and dental materials [25].

Color measurement is usually done by using the CIELAB color system [14]. CIE L*a*b system is prevalent, providing a standardized technique with helpful analysis of ΔE* values accurately. This system can define small color changes accurately and have many advantages, including objectivity, repeatability, and sensitivity [21]. Selecting the CIEDE 2000 color difference formula (ΔE_00_) that was used in this study as it could create a calculation of single-number shade pass or fail in evaluating minor to medium color discrepancies that are more sensitive than the previous CIE L*a*b system.

Surface roughness refers to the finer irregularities of the surface texture that refers to the action of the production process or the material’s features [8]. Currently, several available methods are present to measure the surface texture of any material, including contact stylus tracing, scanning electron microscopy, and atomic force microscopy. Contact stylus tracing was used in the current study because it was fast, simple, and reliable for the comparative assessment of surface roughness properties of both tested single-shade composite resins [26]. Atomic force microscopy (AFM) is a technique for analyzing the topography of the surface. It is an effective technique for characterizing nanoparticles and nanomaterials because it offers qualitative and quantitative information on several physical properties such as size, shape, surface texture, and roughness with a demonstrating image for any surface type, including polymers, ceramics, composites, glass, and biological materials [27].

Regarding color stability, the specimens immersed in the coffee solution reported a more significant color change when compared to the specimens immersed in distilled water. This result could be due to the adsorption and absorption of the yellow stains, which have low polarity. This low polarity of yellow stain can penetrate deeper layers of resin composite [21], in agreement with many studies [4, 16]. On the opposite side, a study found an acceptable color change after immersion in coffee for 48 h E < 3.3; this may be due to differences in immersion solution preparation methods and concentration [28].

Perceptibility and acceptability thresholds determine if a color variation is perceptible and whether it is acceptable or not. The current study's perceptibility threshold (ΔE_00_) was set at 0.8. In contrast, the 50:50% acceptability threshold (ΔE_00_) was 1.8 [14]. In our study, it was clear that the perceptibility threshold values for all groups were higher than 0.8, as shown in Table 2 and Fig. 1. Moreover, the acceptability threshold values were higher than 1.8 after 14 days for all groups.

Group O2 and V2 demonstrated unacceptable color change after 14 days of immersion in distilled water which was consistent with a study that had an unacceptable color change of resin composite after immersion in distilled water for five days [21]. Moreover, it has been reported that the water absorption of composite resins reaches its highest level in 7–60 days [16]. In contrast to Farah and Elwi, who found that immersion in distilled water for seven days resulted in imperceptible color changes (ΔE ≤ 1) [29].

Nanohybrid (Venus Pearl) composite was more color unstable than nano-filled composite (Omnichroma). According to the data provided by the manufacturer (Kulzer GmbH) who claimed that, Venus Pearl with novel low shrinkage composition of tricyclodecane (TCD)-urethane monomer, which is characterized by big molecular size that demonstrate good chemical stability [3]. Nanohybrid (Venus Pearl) contains tricyclodecane TCD urethane-based monomer, giving high resistance to discoloration [3]. But lower filler content and presence of nanoclusters could be the reason for the less color resistance in comparison to the nanofilled resin composite (Omnichroma) [8, 9].

Both resin composite materials exhibited statistically significant difference behavior regarding surface roughness at baseline. The O groups showed superior surface smoothness than the V groups, which could be related to the smaller filler size 4 and higher filler loading [30], as mentioned in Table 1. After one day, groups O2 and V2 were significantly the lowest, followed by group O1. While group V2 was significantly the highest. After 14 days, groups O1 and V1 were significantly the highest. At the same time, Group O2 and V2 were significantly the lowest.

A strong and positive correlation between color stability and surface roughness results, as mentioned in (Table 5) was cleared by the ATF images. It was explained by both resin composite materials' structure and chemical composition. Based on the fact that composite resins with smaller filler sizes exhibit smoother surface properties [31] and less color change [4].

The mean color values and surface roughness after 14 days were the highest for both Groups O1 and V1. It could be due to increased interaction between the resin and the chemicals. More water penetration inside the resin with staining substances of the coffee solution occurred. These conclusions agree with many previous studies [4, 9, 16, 21].

It was stated that when inorganic fillers deboned from the resin matrix, this may leave voids, resulting in surface roughness, forming a surface susceptible to external stains [8, 32]. Additionally, the resin matrix plays an essential role in staining susceptibility [21, 33, 34]. Many studies stated that the ability of resin composite to discolor depends on the resin matrix's hydrophilicity and the material's ability to absorb water [32, 35]. Both materials have a matrix composition based on triethylene glycol dimethacrylate (TEGDMA) and urethane dimethacrylate (UDMA). It was reported that TEGDMA monomer is responsible for color change due to high water absorption and increased coloration [4, 16]. In agreement with a study where the most color change was related to the nanofilled single shade resin composite (Omnichroma) after immersion in coffee for one day in comparison to multi-shade resin composite that could be due to TEGDMA in its composition [4]. Different opposite studies' findings stated no correlation between color and roughness [36].

Although the present study confirmed the detrimental effects of tested solutions on single-shade resin composite material, our study has several limitations. Similarly to other in vitro studies, there are factors affecting the restorations in the oral cavity: microbiota, saliva circulation, temperature, and pH changes. Therefore, the oral cavity could not be imitated precisely [16].

## Conclusions

Based on the results gained from this study, we concluded that;

- 1- Type of resin composite, and immersion periods have a noticeable effect on color stability and surface roughness of single shade resin composite.
- 2- The single-shade resin composite tested showed "extremely" high perceptibility and acceptability threshold values and surface roughness even with distilled water.
- 3- More studies are needed to dig in-depth into the behavior of such materials.

## Data Availability

The datasets used and analyzed during the current study are available from the corresponding author upon reasonable request.

## Abbreviations

ΔE: Color changes
Ra: Roughness values
AFM: Atomic Force Microscope
CIE: Commission International De L’éclairage system
SEM: Scanning electron microscope
REC: The Research Ethics Committees
TEGDMA: Triethylene glycol dimethacrylate
UDMA: Urethane dimethacrylate
TCD: Tricyclodecane
